# Influence Diagnostic Methods in the Poisson Regression Model with the Liu Estimator

**DOI:** 10.1155/2021/4407328

**Published:** 2021-09-08

**Authors:** Aamna Khan, Muhammad Amanullah, Muhammad Amin, Randa Alharbi, Abdisalam Hassan Muse, M. S. Mohamed

**Affiliations:** ^1^Department of Statistics, Bahauddin Zakariya University, Multan, Pakistan; ^2^Department of Statistics, University of Sargodha, Sargodha, Pakistan; ^3^Department of Statistics, Faculty of Science, University of Tabuk, Tabuk, Saudi Arabia; ^4^Department of Mathematics (Statistics Option) Programme, Pan African University, Institute of Basic Science, Technology and Innovation (PAUSTI), Nairobi 6200-00200, Kenya; ^5^Department of Mathematics, College of Science, Taif University, P.O. Box 11099, Taif 21944, Saudi Arabia

## Abstract

There is a long history of interest in modeling Poisson regression in different fields of study. The focus of this work is on handling the issues that occur after modeling the count data. For the prediction and analysis of count data, it is valuable to study the factors that influence the performance of the model and the decision based on the analysis of that model. In regression analysis, multicollinearity and influential observations separately and jointly affect the model estimation and inferences. In this article, we focused on multicollinearity and influential observations simultaneously. To evaluate the reliability and quality of regression estimates and to overcome the problems in model fitting, we proposed new diagnostic methods based on Sherman–Morrison Woodbury (SMW) theorem to detect the influential observations using approximate deletion formulas for the Poisson regression model with the Liu estimator. A Monte Carlo method is done for the assessment of the proposed diagnostic methods. Real data are also considered for the evaluation of the proposed methods. Results show the superiority of the proposed diagnostic methods in detecting unusual observations in the presence of multicollinearity compared to the traditional maximum likelihood estimation method.

## 1. Introduction

Nowadays, there are several distributions available in the literature that can be used to remove noise and then predict data. Similarly, there is a persistent record of concern in modeling count data which has several applications in biosciences and other disciplines [1–4]. The focus of this effort is on dealing with the issues that occur after modeling the count data. For the prediction and analysis of count data, it is valuable to study the factors that influence the performance of the model and the decision based on the analysis of that model. Considering the suitable statistical modeling, when the dependent variable is count data, one of the most used statistical models is the Poisson regression model (PRM). For accurate statistical inferences, the standard ordinary least square (OLS) regression sets some important assumptions related to the model's errors [5]. Generally, numerous problems may arise when a count variable model is estimated using the OLS method, because of the level of noise. For the analysis of count data, PRM provides the most relevant results. According to McCullagh and Nelder [6], the PRM belongs to the family of GLM. The maximum likelihood ML estimation method is used to estimate the PRM estimates instead of the OLS method.

In the PRM, when the explanatory variables are linearly correlated, then the ML method is very sensitive [7]. Some biased estimators were introduced in the literature to handle the multicollinearity, i.e., Stein, ridge, Lasso, regularization, and Liu estimators; see [1, 3] and [8–10] for more details. The most popular one is the ridge estimator, but it has some limitations, i.e., selecting the ridge parameter, where the ridge rule is based on two normal distributions. It is a shrinkage rule because it depends on the slope. In contrast, Lasso is based on the slope and the intercept‬. The best choice is to adopt a Liu estimator to avoid the hindrances of the ridge estimator. The Liu estimator is an ace in this regard as it avoids the disadvantages of the ridge estimator [10], where the main advantage of the ridge is easy to use, and it can be written in the explicate and the objective formulas. In the literature, various studies are available for the PRM to overcome the presence of collinearity [7, 11–16].

To evaluate the reliability and quality of regression estimates and to overcome the problems in model fitting, diagnostic techniques have been developed. Although regression diagnostics have been developed methodologically and theoretically for linear regression models together with multicollinearity (see [17–24]), some studies about the influence diagnostics in the GLM with uncorrelated explanatory variables are available in the literature. Pregibon [25] proposed the influence diagnostics for logistic regression using the one-step methods. For further discussion on influential diagnostics about GLM, see [26–32].

Influence diagnostics in the GLM with correlated explanatory variables is very limited. Özkale et al. [33] proposed the first study on influence diagnostics for logistic ridge regression. Amin et al. [34] worked on the influence diagnostics for the gamma ridge regression model. Khan et al. [35] assessed the performance of influence diagnostics in the PRM with a ridge estimator. Recently, Khan et al. [36] examined the superiority of influence diagnostics in the PRM with two-parameter estimator and, further, Amin et al. [37] discussed the influence diagnostics for the inverse Gaussian ridge regression model.

The available literature showed that no study in the GLM is available for influence diagnostics with the Liu estimator. Though, the Poisson Liu regression (PLR) diagnostics have got no thoughtful attention up till now. Thus, our present work is an effort to fill this gap. So, in the present work, we proposed diagnostic methods for the PRM under the Liu estimator, which prove to be the competed method.

The remaining of the study is organized as follows: we focused on the formulation of influence diagnostic measures for the PRM under the Liu estimator (LE). Next, in Sections 4 and 5, we conducted a Monte Carlo study using two, four, and six independent variables to examine the level of detection percentage of newly developed diagnostic measures and, finally, we proved the efficacy of proposed measures with the help of real world application.

### 1.1. Model Specification and Estimator

Suppose the model can be written as

(1) $$\begin{array}{c} y=X\beta +ɛ, \end{array}$$

where *y*={*y*_*i*_ : *i*=1,2,…, *n*} are the observation, *X*={*x*_*ij*_ : *i*=1,2,…, *n*, *j*=1,2,…, *p*} is a matrix, *β*={*β*_*i*_ : *i*=1,2,…, *p*} are the unknown parameters, and *ɛ* ~ *N*_*n*_(0, *Iσ*^2^) with *ɛ*_*i*_ and *ɛ*_*j*_(*i* ≠ *j*) being independent. We assume the observation is the result of the integration form (*Xβ*) and try to solve this problem by finding differentiation matrix. The PRM is applicable for real data, especially when the response variable *y*_*i*_ often comes in the form of count data that are known. Let *y*_*i*_ follow a Poisson distribution with *μ*_*i*_, as its parameter. The probability mass function for PRM is used to describe the relationship when *y*_*i*_, the response variable occurs as count data.

(2) $$\begin{array}{c} f\left(y_{i};\mu_{i}\right)=\frac{e^{-\mu_{i}}\mu_{i}^{y_{i}}}{y_{i}!}\mu_{i}>0,\;y=0,1,2,\ldots . \end{array}$$

The PRM belongs to the GLM with log link function as

(3) $$\begin{array}{c} \ln\left(\hat{\mu }\right)=b_{0}+b_{1}x_{1}+b_{2}x_{2}+\cdots +b_{p}x_{p}, \end{array}$$

where *b*_0_ is the intercept and *b*_1_, *b*_2_,…, *b*_*p*_ are the set of coefficients. The estimated mean function is defined by ${\hat{\mu }}_{i}=\exp\left(x_{i}^{\prime }\beta \right)$.

Here *x*_*i*_ is the *i*^th^ row of independent variable *X*_*n*×*p*_ and *β*_*p*×1_ of coefficients, where *p* represents the number of explanatory variables.

Assume that all *y*_*i*_ are independent; then, the joint log-likelihood is defined as

(4) $$\begin{array}{c} l\left(\mu ;y_{i}\right)=\sum_{i=1}^{n}\left(y_{i}\ln\left(\exp\left(x_{i}^{\prime }\beta \right)\right)-\exp\left(x_{i}^{\prime }\beta \right)-\ln\left(\prod_{i=1}^{n}y_{i}!\right)\right), \end{array}$$

For finding the best value of *β*, we have to solve the following relation:

(5) $$\begin{array}{c} \frac{\partial l\left(\mu ;y_{i}\right)}{\partial \beta }=0. \end{array}$$

Since the systems of equations are nonlinear, so the MLE with iterative reweighted least-squared (IRLS) algorithm is used to estimate the regression coefficients as explicit formulas:

(6) $$\begin{array}{c} {\hat{\beta }}_{\text{ML}}={\left(X^{\prime }\hat{W}X\right)}^{-1}X^{\prime }\hat{W}\hat{z}, \end{array}$$

where $\hat{W}=\text{diag}\left({\hat{\mu }}_{1},{\hat{\mu }}_{2},\ldots ,{\hat{\mu }}_{n}\right)$ and ${\hat{z}}_{i}=\log\left({\hat{\mu }}_{i}\right)+\left(y_{i}-{\hat{\mu }}_{i}/{\hat{\mu }}_{i}\right)$.

In the presence of multicollinearity, the $X^{\prime }\hat{W}X$ matrix becomes ill conditioned, and because of this problem, it gets complicated to draw effective inferences. To overcome these effects of multicollinearity, we use the generalization of Liu [6] to define PLRE.

(7) $$\begin{array}{c} {\hat{\beta }}_{d}={\left(X^{\prime }\hat{W}X+I\right)}^{-1}\left(X^{\prime }\hat{W}X+dI\right){\hat{\beta }}_{\text{ML}}, \end{array}$$

where 0 ≤ *d* ≤ 1. Here, the important step is selecting shrinkage parameter *d* as the optimal value of *d* which affects the performance of PLRE. Furthermore, if *d*=1, then ${\hat{\beta }}_{\text{ML}}={\hat{\beta }}_{d}$. Recently, Qasim et al. [38] recommended the optimum Liu parameter for the Liu estimator in the PRM as

(8) $$\begin{array}{c} {\hat{d}}_{1}=\max\left(0,\min\left(m_{j}\right)\right),\;j=1,2,\ldots ,p,\\ {\hat{d}}_{2}=\max\left(0,\min\left(h_{j}\right)\right), \end{array}$$

where $m_{j}=\left({\hat{\alpha }}_{j}^{2}-1/\max\left(1/{\hat{\lambda }}_{j}\right)+{\hat{\alpha }}_{j}^{2}\right)$ and $h_{j}=\left({\hat{\alpha }}_{j}^{2}-1/\max\left(1/{\hat{\lambda }}_{j}\right)+{\hat{\alpha }}_{\max}^{2}\right)$ and where *α*_*j*_^2^ is the *j*^th^ the element of *γβ* and the columns of orthogonal matrix *γ* represent the eigenvectors of $X^{t}\hat{W}X$ matrix, such that $X^{t}\hat{W}X=\gamma^{t}\Lambda \gamma$, where Λ=diag(*λ*_1_,…, *λ*_*p*_).

## 2. The PRM Diagnostics

### 2.1. Hat Matrix, Leverage, and Residuals for the PRM

Hat matrix *H* is a common measure used to compute leverages. According to Davison and Tsai [39], the hat matrix *H* in the PRM is

(9) $$\begin{array}{c} H={\hat{W}}^{1/2}X{\left(X^{\prime }\hat{W}X\right)}^{-1}X^{\prime }{\hat{W}}^{1/2}. \end{array}$$

The diagonal elements of *H* are interpreted as leverages, i.e., *h*_*ii*_=diag(*H*). For the computation of regression diagnostic measures, residuals play the most important role (Belsley et al. [18]). Let *χ*_*i*_ symbolize the Pearson residual, so for the case of PRM, we defined it as

(10) $$\begin{array}{c} \chi_{i}=\frac{y_{i}-\exp\left(x_{i}^{\prime }{\hat{\beta }}_{\text{ML}}\right)}{\sqrt{\exp\left(x_{i}^{\prime }{\hat{\beta }}_{\text{ML}}\right)}}, \end{array}$$

Similarly, we find the standardized Pearson residual as

(11) $$\begin{array}{c} \chi_{i}^{\prime }=\frac{\chi_{i}}{\sqrt{\left(1-h_{ii}\right)}}. \end{array}$$

Another useful residual that proves to be of great help for detecting unusual observations is termed as the deviance residual. The *i*^th^ deviance residual for the PRM is defined by

(12) $$\begin{array}{c} d_{i}=\text{sign}\left(y_{i}-\exp\left(x_{i}^{\prime }{\hat{\beta }}_{\text{ML}}\right)\right)\sqrt{2\left[y_{i}\log\left(\frac{y_{i}}{\exp\left(x_{i}^{\prime }{\hat{\beta }}_{\text{ML}}\right)}\right)-\left(y_{i}-\exp\left(x_{i}^{\prime }{\hat{\beta }}_{\text{ML}}\right)\right)\right]}, \end{array}$$

where the sign is the sign function [31].

### 2.2. Influence Diagnostic Methods

Pregibon [25] was the first to work on logistic regression diagnostics tool and proposed the influence diagnostic measures using one-step approximations. The proposed influence diagnostics take account of Cook's distance, change in deviance, and change in Pearson *χ*^2^. For PRM Cook's distance, *C*_*i*_ is suggested as

(13) $$\begin{array}{c} C_{i}=\frac{{\left({\hat{\beta }}_{\text{ML}}-{\hat{\beta }}_{\text{ML}\left(i\right)}\right)}^{\prime }X^{\prime }\hat{W}X\left({\hat{\beta }}_{\text{ML}}-{\hat{\beta }}_{\text{ML}\left(i\right)}\right)}{\left(p+1\right)}. \end{array}$$

The *i*^th^*C*_*i*_ measures the overall change in the fitted model when the *i*^th^ observation is deleted from the model. The one-step approximation for the expression $\left({\hat{\beta }}_{\text{ML}}-{\hat{\beta }}_{\text{ML}\left(i\right)}\right)$ is defined as

(14) $$\begin{array}{c} \Delta {\hat{\beta }}_{\text{ML}i}=\left({\hat{\beta }}_{\text{ML}}-{\hat{\beta }}_{\text{ML}\left(i\right)}\right)=\frac{{\left(X^{\prime }\hat{W}X\right)}^{-1}x_{i}{\hat{W}}_{ii}^{1/2}\chi_{i}}{\left(1-h_{ii}\right)}, \end{array}$$

where ${\hat{W}}_{ii}$ are the *i*^th^ diagonal elements of weight matrix after the removal of *i*^th^ observation. Furthermore, (13) can also be approximated as

(15) $$\begin{array}{c} C_{i}=\frac{\chi_{i}^{\prime 2}}{\left(p+1\right)}\frac{h_{ii}}{\left(1-h_{ii}\right)}. \end{array}$$

Hardin and Hilbe [40] suggested the cut point for detecting the unusual observations in GLM as (4/(*n* − 1)); this process is used to specify the window in GLM.

Pregibon [25] suggested change in Pearson *χ*^2^ as another influence diagnostic measure to detect the influential observations. Applying one-step approximation, we defined Δ*χ*_*i*_^2^ as

(16) $$\begin{array}{c} \Delta \chi_{i}^{2}=\chi_{\left(i\right)}^{2}-\chi_{0}^{2}=\frac{\chi_{i}^{2}}{1-h_{ii}}, \end{array}$$

where *χ*_0_^2^ is used to represent the squared Pearson residuals of the complete data set and *χ*_*i*_^2^ signifies the squared Pearson residuals of the data set without the *i*^th^ observation, respectively. This statistic is employed to study the effect of *i*^th^ observation on the goodness of fit of the model and the estimates. On similar grounds, Pregibon [25] suggested that another statistic for measuring the impact of *i*^th^ observation on the goodness of fit of a model is the change in deviance statistic. The one-step linear approximation for change in deviance statistic is defined as

(17) $$\begin{array}{c} \Delta d_{i}^{2}=d_{\left(i\right)}^{2}-d_{0}^{2}=d_{i}^{2}+\frac{\chi_{i}^{2}h_{ii}}{1-h_{ii}}, \end{array}$$

where for complete data set *d*_0_ is used to represent the squared deviance residuals and the squared deviance residual *d*_(*i*)_ are found after the removal of *i*^th^ observation, respectively. We suggested a simplified form of equation (17) by replacing *χ*_*i*_^2^ by *d*_*i*_^2^ as

(18) $$\begin{array}{c} \Delta d_{i}^{2}=\frac{d_{i}^{2}}{1-h_{ii}}. \end{array}$$

The cut-off value for change in deviance statistic is 3.84 to detect the unusual observations [25].

The difference of fits (DFFITS)  suggested by Belsley et al. [18] is another common influence measure. After deleting the *i*^th^ observation, DFFITS  assesses the change in fit of model. For GLM, it is given as

(19) $$\begin{array}{c} {\text{DFFITS}}_{i}=\frac{{\hat{\mu }}_{i}-{\hat{\mu }}_{i\left(i\right)}}{\sqrt{h_{ii}}}, \end{array}$$

where ${\hat{\mu }}_{i}$ is used to represent the predicted regressand of complete data set and ${\hat{\mu }}_{i\left(i\right)}$ represents the predicted regressand after deleting the *i*^th^ case. Furthermore, it can also be written as

(20) $$\begin{array}{c} {\text{DFFITS}}_{i}=\frac{\sqrt{W_{ii}}x_{i}^{\prime }\left({\hat{\beta }}_{\text{ML}}-{\hat{\beta }}_{\text{ML}\left(i\right)}\right)}{\sqrt{h_{ii}}}. \end{array}$$

By using the SMW theorem, (20) is retransformed as

(21) $$\begin{array}{c} {\text{DFFITS}}_{i}=\left|t_{i}\right|\sqrt{\frac{h_{ii}}{1-h_{ii}}}, \end{array}$$

where $t_{i}=\chi_{i}^{\prime }\sqrt{\left(n-p-1/n-p-\chi_{i}^{\prime 2}\right)}$ is termed as the jackknife Pearson residual and ${\text{DFFITS}}_{i}>2\sqrt{\left(p+1\right)/n}$ shows that the *i*^th^ observation as influential. The second matrix will be introduced in the next section.

## 3. Influence Measures in Poisson Liu Regression Model (PLRM)

### 3.1. Hat Matrix, Leverages, and Residual in PLRM

Hat matrix *H*_*d*_ for the PLRM is defined as

(22) $$\begin{array}{c} H_{d}=X{\hat{W}}^{1/2}{\left(X^{\prime }\hat{W}X+I\right)}^{-1}\left(X^{\prime }\hat{W}X+dI\right){\left(X^{\prime }\hat{W}X\right)}^{-1}W^{1/2}X^{\prime }. \end{array}$$

The leverages are the Liu hat diagonals that proved helpful in detecting influential cases with some modifications. As for *d* > 0, *h*_*di*_ < *h*_*i*_ for *i*=1,2,…, *n* and as *d* increases, *h*_*di*_ decreases monotonically.

Using the Liu estimator, the Pearson residuals for PLRM are defined as

(23) $$\begin{array}{c} \chi_{di}=\frac{y_{i}-\exp\left(x_{i}^{\prime }{\hat{\beta }}_{d}\right)}{\sqrt{\exp\left(x_{i}^{\prime }{\hat{\beta }}_{d}\right)}}. \end{array}$$

The standardized form of Pearson residuals with multicollinear independent variables is given as

(24) $$\begin{array}{c} \chi_{di}^{\prime }=\frac{\chi_{di}}{\sqrt{\left(1-h_{dii}\right)}}. \end{array}$$

### 3.2. Influence Diagnostics for PLRM

The approximate case deletion formulas using SMW theorem [41] are found for the identification of influential observations.

**Theorem 1 .**

After the deletion of *i*^th^ row from ${\hat{\beta }}_{d}$, we write ${\hat{\beta }}_{d\left(i\right)}$ as

(25) $$\begin{array}{c} {\hat{\beta }}_{d\left(i\right)}={\left[X_{\left(i\right)}^{\prime }\hat{W}X_{\left(i\right)}+I\right]}^{-1}\left[X_{\left(i\right)}^{\prime }\hat{W}X_{\left(i\right)}+dI\right]{\hat{\beta }}_{\text{ML}\left(i\right)}, \end{array}$$

where *X*_(*i*)_ represents the *X* matrix without the *i*^th^ row. Using the SMW theorem, we approximated ${\hat{\beta }}_{d\left(i\right)}$.

**Proof**

Letting $K=\sqrt{\hat{W}}X,v=\sqrt{\hat{W}}z,\text{ and }s=y-\hat{\mu }$, then ${\hat{\beta }}_{\text{ML}}$ and ${\hat{\beta }}_{d}$ stated by (6) and (7) become

(26) $$\begin{array}{c} {\hat{\beta }}_{\text{ML}}={\left(K^{\prime }K\right)}^{-1}K^{\prime }v,\\ {\hat{\beta }}_{d}={\left(K^{\prime }K+I\right)}^{-1}\left(K^{\prime }K+d{\hat{\beta }}_{\text{ML}}\right). \end{array}$$

Let ${\hat{\beta }}_{\text{ML}\left(i\right)}$ and ${\hat{\beta }}_{d\left(i\right)}$ represent the ML and PLRE of *β* after deleting the *i*^th^ observation, respectively. Thus, we have

(27) $$\begin{array}{c} {\hat{\beta }}_{\text{ML}\left(i\right)}={\left(K_{\left(i\right)}^{\prime }K_{\left(i\right)}\right)}^{-1}X_{\left(i\right)}^{\prime }s_{\left(i\right)},\\ {\hat{\beta }}_{d\left(i\right)}={\left(K_{\left(i\right)}^{\prime }K_{\left(i\right)}+I\right)}^{-1}\left(K_{\left(i\right)}^{\prime }K_{\left(i\right)}+d{\hat{\beta }}_{\text{ML}\left(i\right)}\right). \end{array}$$

With the help of SMV theorem, ${\hat{\beta }}_{\text{ML}\left(i\right)}$ can be improved as

(28) $$\begin{array}{c} {\hat{\beta }}_{\text{ML}\left(i\right)}=\left[{\left(K^{\prime }K\right)}^{-1}+\frac{{\left(K^{\prime }K\right)}^{-1}k_{i}^{\prime }k_{i}{\left(K^{\prime }K\right)}^{-1}}{1-m_{i}}\right]\left(X^{\prime }s-x_{i}s_{i}\right), \end{array}$$

where $k_{i}^{\prime }=\sqrt{{\hat{W}}_{ii}}x_{i}^{\prime }$ is the *i*^th^ row vector of the *K* matrix and *m*_*i*_=*k*_*i*_(*K*′*K*)^−1^*k*_*i*_′ solves the first part of R.H.S of (27)

(29) $$\begin{array}{c} {\left(K_{\left(i\right)}^{\prime }K_{\left(i\right)}+I\right)}^{-1}={\left[\left(K^{\prime }K+I\right)-k_{i}^{\prime }k_{i}\right]}^{-1}={\left(K^{\prime }K+I\right)}^{-1}+\frac{{\left(K^{\prime }K+I\right)}^{-1}k_{i}^{\prime }k_{i}{\left(K^{\prime }K+I\right)}^{-1}}{1-m_{di}}, \end{array}$$

where *m*_*di*_=*k*_*i*_(*K*′*K*+*I*)^−1^*k*_*i*_′. We also have

(30) $$\begin{array}{c} {\left(K_{\left(i\right)}^{\prime }K_{\left(i\right)}+I\right)}^{-1}\left(K_{\left(i\right)}^{\prime }K_{\left(i\right)}+d{\hat{\beta }}_{\text{ML}}\right)={\left[\left(K^{\prime }K+I\right)-k_{i}^{\prime }k_{i}\right]}^{-1}\left(K^{\prime }K+d{\hat{\beta }}_{\text{ML}}-k_{i}^{\prime }k_{i}\right)\\ ={\left(K^{\prime }K+I\right)}^{-1}\left(K^{\prime }K+d{\hat{\beta }}_{\text{ML}}\right)+\frac{{\left(K^{\prime }K+I\right)}^{-1}k_{i}^{\prime }k_{i}{\left(K^{\prime }K+I\right)}^{-1}\left(K^{\prime }K+d{\hat{\beta }}_{\text{ML}}\right)}{1-m_{di}}-\frac{{\left(K^{\prime }K+I\right)}^{-1}k_{i}^{\prime }k_{i}}{1-m_{di}}. \end{array}$$

Now,

(31) $$\begin{array}{c} {\hat{\beta }}_{d\left(i\right)}={\left(K^{\prime }K+I\right)}^{-1}\left(K^{\prime }K+d{\hat{\beta }}_{\text{ML}}\right)-\frac{{\left(K^{\prime }K+I\right)}^{-1}k_{i}^{\prime }}{1-m_{di}}\left(\frac{s_{i}}{\sqrt{{\hat{W}}_{ii}}}-k_{i}{\left(K^{\prime }K+I\right)}^{-1}\left(K^{\prime }K+d{\hat{\beta }}_{\text{ML}}\right)\right)\\ ={\hat{\beta }}_{d}-\frac{{\left(K^{\prime }K+I\right)}^{-1}k_{i}^{\prime }}{1-m_{di}}\left(\frac{s_{i}}{\sqrt{{\hat{W}}_{ii}}}-k_{i}{\hat{\beta }}_{d}\right)\\ ={\hat{\beta }}_{d}-\frac{{\left(X^{\prime }\hat{W}X+I\right)}^{-1}x_{i}^{\prime }\sqrt{{\hat{W}}_{ii}}\chi_{di}}{1-m_{di}}\\ {\hat{\beta }}_{d}-{\hat{\beta }}_{d\left(i\right)}=\frac{{\left(X^{\prime }\hat{W}X+I\right)}^{-1}x_{i}^{\prime }\sqrt{{\hat{W}}_{ii}}\chi_{di}}{1-m_{di}}. \end{array}$$

Hence, the theorem is completed.

Following [42] for the PLRE, the Cook's distance is redefined as

(32) $$\begin{array}{c} C_{di}=\frac{{\left({\hat{\beta }}_{d}-{\hat{\beta }}_{d\left(i\right)}\right)}^{\prime }\left(X^{\prime }\hat{W}X\right)\left({\hat{\beta }}_{d}-{\hat{\beta }}_{d\left(i\right)}\right)}{\left(p+1\right)}. \end{array}$$

The *i*^th^ observation is considered as influential if the distance between ${\hat{\beta }}_{d\left(i\right)}$ and ${\hat{\beta }}_{d}$ is larger. Another version can be expressed as

(33) $$\begin{array}{c} C_{di}=\frac{1}{\left(p+1\right)}{\left[{\hat{\beta }}_{d}-{\hat{\beta }}_{d\left(i\right)}\right]}^{\prime }\left(X^{\prime }\hat{W}X+I\right){\left(X^{\prime }\hat{W}X+dI\right)}^{-1}\times \left(X^{\prime }\hat{W}X\right){\left(X^{\prime }\hat{W}X+dI\right)}^{-1}\left(X^{\prime }\hat{W}X+I\right)\left[{\hat{\beta }}_{d}-{\hat{\beta }}_{d\left(i\right)}\right]. \end{array}$$

Using the Liu estimator, we defined the change in Pearson chi-square as

(34) $$\begin{array}{c} \Delta \chi_{di}^{2}=\Delta \chi_{d\left(i\right)}^{2}=\Delta \chi_{d0}^{2}=\frac{1}{1-h_{dii}}\left[\frac{{\left(y_{i}-{\hat{\mu }}_{di}\right)}^{2}}{{\hat{\mu }}_{di}}\right], \end{array}$$

where the squared Liu Pearson residuals *χ*_*d*0_^2^ are used to represent the complete data set and *χ*_*d*(*i*)_^2^ computed without *i*^th^ observation. Correspondingly, with Liu estimator, we formulated the change in deviance statistic as

(35) $$\begin{array}{c} \Delta d_{d}^{2}=d_{d\left(i\right)}^{2}-d_{d0}^{2}=d_{di}^{2}+\frac{\chi_{di}^{2}h_{dii}}{1-h_{dii}}, \end{array}$$

where *d*_*d*0_^2^ and *d*_*d*(*i*)_^2^ represent the squared Liu deviance residuals with complete data and the squared Liu deviance residuals computed without *i*^th^ observation, and

(36) $$\begin{array}{c} d_{di}=s_{i}\sqrt{2\left(y_{i}\log\left(\frac{y_{i}}{\exp\left(x_{i}^{\prime }{\hat{\beta }}_{d}\right)}\right)-\left(y_{i}-\exp\left(x_{i}^{\prime }{\hat{\beta }}_{d}\right)\right)\right)}, \end{array}$$

where *s*_*i*_ is the sign function of $\left(y_{i}-\exp\left(x_{i}^{\prime }{\hat{\beta }}_{d}\right)\right)$.

Following (19), we give the DFFITS for PLRM as

(37) $$\begin{array}{c} {\text{DFFITS}}_{di}=\frac{{\hat{\mu }}_{di}-{\hat{\mu }}_{di\left(i\right)}}{\sqrt{h_{dii}}}=\frac{\sqrt{W_{ii}}x_{i}^{\prime }\left({\hat{\beta }}_{d}-{\hat{\beta }}_{d\left(i\right)}\right)}{\sqrt{h_{dii}}}, \end{array}$$

where ${\hat{\mu }}_{d0}$ and ${\hat{\mu }}_{d\left(i\right)}$ represent the predicted regressand of the complete data set and predicted regressand after deleting the *i*^th^ case.

Using the SMW theorem, we simplified (37) as

(38) $$\begin{array}{c} {\text{DFFITS}}_{di}=\left|t_{di}\right|\sqrt{\frac{h_{dii}}{1-h_{dii}}}, \end{array}$$

where $t_{di}=\chi_{di}^{\prime }\sqrt{\left(n-p^{\prime }/n-p-\chi_{di}^{\prime 2}\right)}$ is the *i*^th^ Pearson Jackknife residual with Liu estimator.

## 4. Simulation Study

In this section, we summarize the results of the PRM and the PLRM influence diagnostics using the Monte Carlo simulation scheme. We follow the same simulation scheme used by many researchers to see [43, 44]. The response variable *y* is generated from the Poisson distribution with mean function *μ*_*i*_ as defined by

(39) $$\begin{array}{c} \mu_{i}=\exp\left(\beta_{0}+\beta_{1}x_{i1}+\beta_{2}x_{i2}+\cdots +\beta_{p}x_{ip}\right),\;i=1,2,\ldots ,n. \end{array}$$

We set simulation with *p*=2,4,6 explanatory variables with various sample sizes plus the mild to severe levels of collinearity. We assumed sample sizes *n*=25,50,100,150,200. Moreover, we generated the regressors using the following formula:

(40) $$\begin{array}{c} x_{ij}=\sqrt{\left(1-\rho^{2}\right)}z_{ij}+\rho z_{ip}+1,\;j=1,2,\ldots ,p+1,i=1,2,\ldots ,n. \end{array}$$

We consider the different collinearity levels as *ρ*^2^=0.75, 0.85, 0.95, 0.99, and we assume the arbitrary values of regression coefficients in such a way that ∑_*j*=1_^*p*^*β*_*j*_^2^=1. Now we generated few influential observations in the regressors by using the expression *X*_*ij*_=*X*_*ij*_+*α*_0_, *i*=15 and *j*=1,2,…, *p*, where $\alpha_{0}={\bar{X}}_{j}+6$. All the analyses are performed using the *R* software with 1000 replications.

### 4.1. Results and Discussion

The study results of the calculations of the identification of the unusual observations with LE in the presence of mild to severe multicollinearity are provided in Tables 1–6 with *p*=2,4,  and 6 with defined optimum *d*_1_ and *d*_2_. From Tables 1–3 with *p* = 2, it is clear that performed *C*_*di*_ is good as compared to the *C*_*i*_ method for different sample sizes with multicollinearity. The influence detection of Δ*χ*_*di*_^2^ and Δ*d*_*di*_^2^ methods is identical and performs significantly better than Δ*χ*_*i*_^2^ and Δ*d*_*i*_^2^, respectively. However, it is observed that their performance does not occur in a better way than that of the *C*_*i*_ method for all the combinations of *n*, *p* and *ρ*. Comparable effects are observed on DFFITS_*i*_ method, and it is found that the detection percentage of influential observations by DFFITS_*i*_ method is better than *C*_*i*_, although the performance of DFFITS_*di*_ related to *C*_*di*_ is equally better. Furthermore, as we increased the sample sizes, the percentage of detecting the influential observation of the developed measures equally increases. Moreover, from Tables 4–6, we observed that the newly developed diagnostic measures performed more efficiently with *d*_2_, but *d*_1_ give better detection percentage as compared to *d*_2_.  Furthermore, varying the regressors size affects the functioning of *C*_*di*_ method and DFFITS_*di*_ method, respectively. Δ*χ*_*di*_^2^ and Δ*d*_*di*_^2^ values are larger than Δ*χ*_*i*_^2^ and Δ*d*_*i*_^2^, respectively. Further the changing pattern of sample size and multicollinearity together with their effects are demonstrated explicitly to study the performance of newly developed measures through graphs; see Figures 1, 2, and 3 for defined *d*_1_ and *d*_2_. Considering Figures 1–3, with defined combinations of sample sizes, regressors, and collinearity levels, we clearly observe a positive increase in the performance of newly developed measures.

## 5. Application: English League Football Data

For the illustration of the proposed diagnostic methods, we analyze the football English League data set which is also available in Table 7. The said data comprise *n*=20 observations with one response variable, i.e., the number of won matches (*y*) and *p* = 5 explanatory variables, i.e., the number of yellow cards (*X*_1_), the number of red cards (*X*_2_), goals won (*X*_3_), goals conceded (*X*_4_), and the number of points earned (*X*_5_). Algamal and Alanaz [11] also used this data set. After checking the *χ*^2^, the goodness of fit test found that it is well fitted to the Poisson distribution. The said data are multicollinear as the condition index CI = 31.274.

From Table 8, it is found that all methods commonly identify the 1st observation as the influential observation. Change in chi-square statistic and change in deviance statistic with ML estimator do not detect any of the observation as influential. Furthermore, observation 19^th^ was detected as influential by DFFITS without Liu estimator and by all of the proposed diagnostics.

The effect of deleting the highlighted observations on the estimates of PRM and PLRM is presented in Table 9. We found a maximum change in PRM and PLRM estimates after the removal of the 1^st^ observation that was detected by all selected and proposed measures. The second observation that was identified by just DFFITS_*i*_ and all proposed measures is the 19^th^. After the deletion of detected observations, we found the maximum change on ${\hat{\beta }}_{2}$ and ${\hat{\beta }}_{3}$. After examining these results, it was noted that in the presence of multicollinearity, PLRM diagnostic measures efficiently detect the influential observations. Furthermore, we incorporated index plots to summarize the efficacy of the proposed measures in Figure 4.

## 6. Conclusion

This study introduces diagnostic measures for Poisson Liu regression using biased estimator to handle influential observations and multicollinearity simultaneously in the PRM. As discussed earlier, multicollinearity affects the performance of traditional ML estimator in PRM. Therefore, we adopted the Liu estimator due to its efficient statistical properties to solve multicollinearity and influential observations in PRM. The simulation results support the performance of new diagnostic measures as the detection percentage of ML estimators and the existing measures turn out to be the worst with increasing the sample size, number of regressors, and the level of multicollinearity. The results proved that the suggested measures proved more beneficial for the identification of influential observations together with multicollinearity. Hence, it is suggested that these proposed measures guide the user to handle the issue of multicollinearity with robust estimator support efficiently.

## Figures and Tables

**Figure 1:** Graph of influential observation detection percentages of proposed measures for *p* = 2.

**Figure 2:** Graph of influential observation detection percentages of proposed measures for *p* = 4.

**Figure 3:** Graph of influential observation detection percentages of proposed measures for *p* = 6.

**Figure 4:** Graphical representation of influential observations in English League Football data.

**Table 1:** Influence diagnostics detections (%) with *d*_1_ and *p*=2.

*n*	*ρ* ^2^	*C*_*i*_	Δ*χ*_*i*_^2^	Δ*d*_*i*_^2^	DFFITS_*i*_	*C*_*di*_	Δ*χ*_*di*_^2^	Δ*d*_*di*_^2^	DFFITS_*di*_
25	0.75	79.2	47.5	47.5	96.1	91.8	77	76.9	91.8
	0.85	77.6	42.4	42.4	95.1	91.1	75.7	75.8	90.9
	0.95	79.5	44.9	44.9	95.1	90.2	77.1	77.1	90.2
	0.99	75.6	40	40	94.5	90.3	72.2	72.2	90.3

50	0.75	80.9	37.1	37.1	97	91.9	71	71.1	91.9
	0.85	81	35.9	35.9	97.6	91	70.7	70.5	91
	0.95	79.3	32.6	32.6	97.3	90.8	68.8	68.7	90.8
	0.99	78.5	33.2	33.2	96.1	91.2	68.2	68.1	91.2

100	0.75	89.5	42.2	42.2	98.6	95.9	73.9	73.7	95.9
	0.85	87.5	37.9	37.9	99	94.4	72.8	72.7	94.4
	0.95	86.3	35.7	35.7	97.9	94.8	70.1	70.1	94.8
	0.99	86.9	39.1	39.1	98.4	95.4	74.2	74.4	95.4

150	0.75	91	45	45	99.2	96.1	76.8	76.9	96.1
	0.85	89.1	39.3	39.3	98.7	95.3	72.6	72.6	95.3
	0.95	90.8	38.3	38.3	99.2	96	73	72.9	96
	0.99	88.2	39.7	39.7	99	94.9	71.8	71.8	94.9

200	0.75	91.6	47.4	47.4	99.3	96.5	75.4	75.5	96.5
	0.85	91.4	42.7	42.7	99.1	96.7	73.5	73.5	96.7
	0.95	90.7	41.1	41.1	99.9	95.3	72.5	72.5	95.3
	0.99	93.8	41.3	41.3	99.3	96.8	75.6	75.5	96.8

**Table 2:** Influence diagnostics detections (%) with *d*_1_ and *p*=4.

*n*	*ρ* ^2^	*C*_*i*_	Δ*χ*_*i*_^2^	Δ*d*_*i*_^2^	DFFITS_*i*_	*C*_*di*_	Δ*χ*_*di*_^2^	Δ*d*_*di*_^2^	DFFITS_*di*_
25	0.75	75.9	57	57	94.8	91	82.6	82.6	90.9
	0.85	69.7	48.9	48.9	93.7	87.8	76.4	76.4	87.7
	0.95	67.3	45.6	45.6	93.5	85.4	74.3	74.3	85.3
	0.99	65.7	44.4	44.4	93.9	85.3	74.3	74.2	85.2

50	0.75	78.6	47.8	47.8	97.4	91.5	77.9	77.9	91.4
	0.85	77.8	44.9	44.9	97.7	90.6	77.5	77.4	90.4
	0.95	74.1	38.6	38.6	95.1	88.5	72.6	72.6	88.5
	0.99	71.7	35.8	35.8	95.9	86.7	68.8	68.7	86.7

100	0.75	86.1	50.4	50.4	98.8	94.4	79.4	79.3	94.4
	0.85	84.8	44.6	44.6	97.9	93.8	77.7	77.7	93.8
	0.95	81.5	39.7	39.7	97.6	91.3	72.5	72.3	91.3
	0.99	82.2	40	40	98.5	93.7	75	75	93.7

150	0.75	86.6	49.6	49.6	98.8	94.5	78.2	78.2	94.5
	0.85	87.5	46.7	46.7	98.8	95.3	78.4	78.5	95.3
	0.95	85.8	42.5	42.5	98.6	94.7	74.3	74.2	94.7
	0.99	86.8	41.4	41.4	99.2	94.5	76.3	76.4	94.5

200	0.75	90.1	50.5	50.5	99	96.6	80.1	80.1	96.6
	0.85	89.8	48	48	99.3	96.3	79.3	79.3	96.3
	0.95	87.7	46.9	46.9	99.2	94.8	75.9	75.9	94.8
	0.99	88.1	39.9	39.9	98.8	95.2	73.7	73.7	95.2

**Table 3:** Influence diagnostics detections (%) with *d*_1_ and *p*=6.

*n*	*ρ* ^2^	*C*_*i*_	Δ*χ*_*i*_^2^	Δ*d*_*i*_^2^	DFFITS_*i*_	*C*_*di*_	Δ*χ*_*di*_^2^	Δ*d*_*di*_^2^	DFFITS_*di*_
25	0.75	73.1	54.5	54.5	93.7	88.6	78.1	78.1	88.4
	0.85	72.3	52.6	52.6	93.6	87.4	78.8	78.8	87.4
	0.95	68.4	47	47	93.9	85.9	76.5	76.5	85.7
	0.99	67.4	45.1	45.1	93	84.5	72.4	72.3	84.5

50	0.75	77.3	46.2	46.2	97.2	91.2	76.9	76.9	91.2
	0.85	74	43.2	43.2	96.5	89.8	74.7	74.7	89.8
	0.95	72.4	38.4	38.4	96.7	89.6	71.6	71.5	89.5
	0.99	73.1	35.2	35.2	95.9	87.5	68.5	68.7	87.5

100	0.75	83.8	47	47	98.7	95.1	77.2	77.1	95.1
	0.85	84.1	46.6	46.6	98.3	94.2	78.7	78.7	94.2
	0.95	82	41.9	41.9	97.8	94	75.4	75.4	94
	0.99	81.4	38.4	38.4	98.5	91.6	71.4	71.3	91.6

150	0.75	88.9	51.5	51.5	98.8	95.4	80.3	80.3	95.4
	0.85	86	47.7	47.7	99.1	94.4	78.1	78.2	94.4
	0.95	86.5	42.7	42.7	98.6	94.2	75.2	75.4	94.2
	0.99	83.9	40.3	40.3	98.7	93.6	71.4	71.4	93.6

200	0.75	90.7	50.1	50.1	99.1	95.3	81.2	81.2	95.3
	0.85	88.8	45.8	45.8	99.2	96.9	76.3	76.3	96.9
	0.95	88	44.8	44.8	99.2	95.5	74.7	74.8	95.5
	0.99	87.7	41.9	41.9	99.3	94.4	75.7	75.7	94.4

**Table 4:** Influence diagnostics detections (%) with *d*_2_ and *p*=2.

*n*	*ρ* ^2^	*C*_*i*_	Δ*χ*_*i*_^2^	Δ*d*_*i*_^2^	DFFITS_*i*_	*C*_*di*_	Δ*χ*_*di*_^2^	Δ*d*_*di*_^2^	DFFITS_*di*_
25	0.75	77.7	44.6	44.6	95.4	91.3	75	75	91.3
	0.85	74.6	38.9	38.9	95.1	89.9	73	73	89.9
	0.95	76.8	42.4	42.4	94.5	89.9	74.4	74.6	89.9
	0.99	75.4	40.6	40.6	95.2	90.3	71.3	71.3	90.3

50	0.75	78.2	35.9	35.9	97.6	91.6	68	68	91.5
	0.85	81	34.5	34.5	98	92.6	69.5	69.6	92.6
	0.95	79.1	35.1	35.1	97	90.8	68.9	68.7	90.7
	0.99	80.2	34.3	34.3	97.2	91.5	67.5	67.5	91.5

100	0.75	87.9	40.1	40.1	98.5	94.3	73.1	73.2	94.3
	0.85	86.6	42.3	42.3	98.2	94	72	72	94
	0.95	88.4	37.1	37.1	98.6	94.8	74.2	74.3	94.8
	0.99	88.8	42.3	42.3	98.6	94.1	73.5	73.4	94.1

150	0.75	91.1	46.1	46.1	98.9	96.4	76.1	76.1	96.4
	0.85	90.3	39.2	39.2	99.8	95.6	72.4	72.4	95.6
	0.95	90.2	38.8	38.8	99	95.9	72	72.1	95.9
	0.99	89.8	39.1	39.1	99.2	95.5	74.7	74.7	95.5

200	0.75	93	44.9	44.9	99.3	96.4	75.9	76	96.4
	0.85	93.2	43.6	43.6	99.6	96.6	77.6	77.7	96.6
	0.95	91.9	41.9	41.9	99.2	96.9	73.4	73.4	96.9
	0.99	92.6	40.3	40.3	99.5	96.3	74.3	74.2	96.3

**Table 5:** Influence diagnostics detections (%) with *d*_2_ and *p*=4.

*n*	*ρ* ^2^	*C*_*i*_	Δ*χ*_*i*_^2^	Δ*d*_*i*_^2^	DFFITS_*i*_	*C*_*di*_	Δ*χ*_*di*_^2^	Δ*d*_*di*_^2^	DFFITS_*di*_
25	0.75	72.7	47.5	47.5	94.6	89.1	76.1	76.2	89.1
	0.85	73.5	46.1	46.1	94.7	88.7	77.4	77.4	88.7
	0.95	69.9	41.2	41.2	91.9	86.5	73.7	73.8	86.5
	0.99	70.3	42.5	42.5	94.2	87.6	73.6	73.6	87.6

50	0.75	79.6	40.6	40.6	96.4	91.2	75.1	75.1	91.2
	0.85	76.5	37.1	37.1	97.4	91.2	73.6	73.4	91.2
	0.95	78.9	38.8	38.8	96.8	89.6	74	74	89.6
	0.99	74.4	36.1	36.1	97.7	90.5	71	70.9	90.5

100	0.75	87	45.5	45.5	99.1	95.7	76.2	76.1	95.7
	0.85	84.1	41.2	41.2	97.8	93.7	73.5	73.5	93.7
	0.95	84.3	38.4	38.4	98.4	94.5	73.5	73.5	94.5
	0.99	86	38.3	38.3	98.9	94.5	74.4	74.3	94.5

150	0.75	89.5	46.3	46.3	99.1	95.9	77.3	77.3	95.9
	0.85	89.5	44.4	44.4	99.2	96	77.7	77.6	96
	0.95	89.6	41.9	41.9	99.1	95.8	76.3	76.4	95.8
	0.99	86.8	38.8	38.8	98.4	94.3	71.5	71.5	94.3

200	0.75	90.9	47.3	47.3	98.8	96.4	79.9	79.8	96.4
	0.85	89.3	43.8	43.8	99.2	95.5	76	75.9	95.5
	0.95	89.6	41.5	41.5	99.6	95.5	75.8	75.8	95.5
	0.99	89.6	41.9	41.9	99.1	95.9	72.6	72.7	95.9

**Table 6:** Influence diagnostics detections (%) with *d*_2_ and *p*=6.

*n*	*ρ* ^2^	*C*_*i*_	Δ*χ*_*i*_^2^	Δ*d*_*i*_^2^	DFFITS_*i*_	*C*_*di*_	Δ*χ*_*di*_^2^	Δ*d*_*di*_^2^	DFFITS_*di*_
25	0.75	75.9	57	57	94.8	91	82.6	82.6	90.9
	0.85	69.7	48.9	48.9	93.7	87.8	76.4	76.4	87.7
	0.95	67.3	45.6	45.6	93.5	85.4	74.3	74.3	85.3
	0.99	65.7	44.4	44.4	93.9	85.3	74.3	74.2	85.2

50	0.75	78.6	47.8	47.8	97.4	91.5	77.9	77.9	91.4
	0.85	77.8	44.9	44.9	97.7	90.6	77.5	77.4	90.4
	0.95	74.1	38.6	38.6	95.1	88.5	72.6	72.6	88.5
	0.99	71.7	35.8	35.8	95.9	86.7	68.8	68.7	86.7

100	0.75	86.1	50.4	50.4	98.8	94.4	79.4	79.3	94.4
	0.85	84.8	44.6	44.6	97.9	93.8	77.7	77.7	93.8
	0.95	81.5	39.7	39.7	97.6	91.3	72.5	72.3	91.3
	0.99	82.2	40	40	98.5	93.7	75	75	93.7

150	0.75	86.6	49.6	49.6	98.8	94.5	78.2	78.2	94.5
	0.85	87.5	46.7	46.7	98.8	95.3	78.4	78.5	95.3
	0.95	85.8	42.5	42.5	98.6	94.7	74.3	74.2	94.7
	0.99	86.8	41.4	41.4	99.2	94.5	76.3	76.4	94.5

200	0.75	90.1	50.5	50.5	99	96.6	80.1	80.1	96.6
	0.85	89.8	48	48	99.3	96.3	79.3	79.3	96.3
	0.95	87.7	46.9	46.9	99.2	94.8	75.9	75.9	94.8
	0.99	88.1	39.9	39.9	98.8	95.2	73.7	73.7	95.2

**Table 7:** English League football data.

**Y** (no. of won matches)	**X1** (no. of yellow cards)	**X2** (no. of red cards)	**X3** (goals own)	**X4** (goals conceded)	**X5** (no. of points earned)
30	72	0	33	52	93
26	62	0	26	60	86
23	71	4	39	41	78
22	54	0	42	36	76
23	68	3	44	33	75
18	78	2	29	25	69
17	72	2	44	18	61
12	59	2	48	−7	46
12	52	3	67	−12	46
12	80	0	51	−8	45
12	78	5	64	−17	45
12	72	1	63	−15	44
11	70	2	56	−15	44
12	77	0	63	−13	41
12	56	0	70	−25	41
11	65	2	55	−16	40
11	84	5	68	−28	40
9	67	5	80	−43	34
5	77	1	53	−26	28
6	78	4	69	−40	24

**Table 8:** Influential observations detected using the PRM and the PLRM.

Procedures	PRM	Procedures	PLRM ${\hat{d}}_{1}$
*C*_*i*_	1	*C*_*di*_	1,19
Δ*χ*_*i*_^2^	—	Δ*χ*_*di*_^2^	1,19
Δ*d*_*i*_^2^	—	Δ*d*_*di*_^2^	1,19
DFFITS_*i*_	1,6,14,19	DFFITS_*di*_	1,6,7,8,10,14,15,16,18,19,20

**Table 9:** Absolute change (%) in the estimates after deletion of influential observations.

Estimates	Influential observations					
	1^st^		19^th^		1^st^ and 19^th^	
	PRM	PLRM	PRM	PLRM	PRM	PLRM
${\hat{\beta }}_{0}$	69.1	81.0	27.6	23.0	11.9	52.0
${\hat{\beta }}_{1}$	3944.7	17.8	1448.5	47.2	3341.4	56.8
${\hat{\beta }}_{2}$	510.0	160.4	139.8	54.4	392.3	189.6
${\hat{\beta }}_{3}$	355.4	626.9	77.7	75.7	119.2	485.2
${\hat{\beta }}_{4}$	144.7	50.9	70.5	19.5	13.9	28.4
${\hat{\beta }}_{5}$	58.1	46.2	20.9	10.5	12.2	31.5

## Data Availability

All data are included in the paper with their links.
